The article "Pro-environmental behavior–Renewable energy transitions nexus: Exploring the role of higher education and information and communications technology diffusion" was retracted in 2025. Reasons: an official misconduct investigation; compromised peer review; a compromised editor; unreliable results or conclusions.

# Pro-environmental behavior–Renewable energy transitions nexus: Exploring the role of higher education and information and communications technology diffusion

**DOI:** 10.3389/fpsyg.2022.1010627

**Published:** 2022-10-11

**Authors:** Ma Deshuai, Li Hui, Sana Ullah

**Affiliations:** ^1^School of Marxism, Jilin University, Changchun, China; ^2^Shenzhen Party School, Shenzhen, China; ^3^School of Economics, Quaid-i-Azam University, Islamabad, Pakistan

**Keywords:** pro-environmental behavior, renewable energy transitions, higher education, ICT, China, digitalization

## Abstract

The most accepted solution to deal with the problems of global warming and climate change is to transform the energy sector by moving toward renewable energy. Therefore, the primary focus of the analysis is to examine the role of renewable energy consumption, higher education, and ICT in improving environmental quality and green growth in China. We have employed the quantile ARDL model to obtain the short-and long-run estimates. According to the findings of QARDL, the long-run estimated coefficients of renewable energy consumption and higher education are positively significant in most quantiles. However, in the long run, the estimates attached to ICT are insignificant in the CO_2_ emissions model in most quantiles. On the other hand, the estimates of renewable energy consumption are significantly positive from the 50th quantile and onward in the green growth model, confirming that the higher the renewable energy in the economy, closer it will get to the target of green economic growth. The long-run estimates of higher education and ICT are positively significant at most quantiles in the green growth model. In the short run, renewable energy consumption turned out to be the most critical determinant of CO_2_ emissions and green growth.

## Introduction

Global warming and climate change are mainly the outcomes of a heavy incursion of carbon emissions into the atmosphere due to a rise in anthropogenic activities in recent times (Ozturk and Ullah, 2022). The main cause behind global warming and climate change is the overuse of dirty energy resources, such as coal, oil, and gas, by the nations to support the process of industrialization, urbanization, trade, and other economic activities. According to the International Energy Agency (IEA), the adverse impact of fossil fuels on human health is such that about 6 million people die due to environmental pollution every year, thereby affecting the financial sector and level of investment in the environment sector (Machol and Rizk, 2013). Therefore, generating renewable and alternative energy sources is considered the most vital approach to controlling environmental damage by controlling carbon emissions (Işik, 2010; Sohail et al., 2021). Increasing the role of renewable energy in the economy also lets the economy proliferate without damaging the environment (Işık et al., 2021a,b).

The article "Pro-environmental behavior–Renewable energy transitions nexus: Exploring the role of higher education and information and communications technology diffusion" was retracted in 2025. Reasons: an official misconduct investigation; compromised peer review; a compromised editor; unreliable results or conclusions.

Renewable energy sources are considered sustainable because they continuously grow with their utilization. The energy obtained from solar, hydel, wind, and biomass is renewable energy and is cost-effective and never-ending. In addition, these sources are environmentally friendly and help achieve better environmental quality (Işık, 2013; Ullah et al., 2020). Moreover, the rise in renewable energy consumption can significantly improve the global energy outlook and make result in more sustainable green development. As a result, the developed and developing nations have invested heavily in increasing the generation of renewable energy sources. For instance, after signing the Paris Agreement (2015), India pledged to accelerate the share of renewable energy sources to 40% of the total energy output by 2030. Since renewable energy is the most significant option for developed and developing economies to cope with the issues of energy security and global warming, the focus of policymakers, environmentalists, and empirics has been to investigate the factors that can affect renewable energy consumption.

The demand for renewable energy is subject to the people’s awareness regarding the issues of global warming and energy security. Renewable energy is a key source of environmental sustainability and green growth. Education can significantly affect renewable energy consumption, and making people more aware of environmental degradation is vital in the generation of renewable energy (Mahalik et al., 2021). To promote better environmental quality, the consciousness, abilities, and attitude of the common people and legislators play an important role due to their positive role in promoting renewable energy consumption (Linde, 1994). By contrast, the shortage of human capital or lack of educated and skilled people in the energy sector also impacts environmental sustainability and green growth (Zafar et al., 2020; Li et al., 2022b). Proficient monitoring and energy demand are the factors that can determine the consumer’s education and environmental mindfulness. Moreover, an educated person can better understand the risks involved in investing in renewable energy projects, which would help them make better decisions regarding renewable energy investments (Zafar et al., 2020). On the other hand, the availability of financial capital is crucial to promoting human capital development and improving education standards in the country. As far as the energy sector is concerned, improved training and skills can fulfill the human capital requirement in technology (Lucas et al., 2018). At the same time, based on environmental awareness, citizens can make prudent decisions regarding applying suitable technology and energy-efficient and pro-environment products.

The article "Pro-environmental behavior–Renewable energy transitions nexus: Exploring the role of higher education and information and communications technology diffusion" was retracted in 2025. Reasons: an official misconduct investigation; compromised peer review; a compromised editor; unreliable results or conclusions.

Lack of technology is considered an important hurdle in implementing renewable energy technologies, particularly in less developing economies (Schäfer et al., 2014). Likewise, technological constraints are considered a blockade in the way of developing renewable energy sources, and the inclusion of renewable energy into the energy mix looks more challenging (Ghaffour et al., 2015). Hence, the absence of technical knowledge is the main reason behind fragile energy infrastructures in low-income countries, which makes the transition process from dirty to clean energy sources a difficult one in these economies (Sabyrbekov and Ukueva, 2019). Against this backdrop, it is pertinent to investigate the factor that can help these low-income nations overcome technological impediments. In this regard, the role of information and communications technology (ICT) can prove significant in helping less developing economies overcome technical constraints, which may promote environmental quality and green growth. The use of ICT is more likely to accelerate green growth. Thus, to ensure the maximum generation of green growth, ICT can play a significant role, mainly when they are easily available. Moreover, increased ICT use also helps store the electricity generated through clean energy sources (Usman et al., 2021). Therefore, the overhauling of the energy infrastructure with the help of ICT could prove vital in overcoming the technological shortcomings that hinder the development of renewable energy transition. Furthermore, ICT diffusion aims to reduce renewable energy production costs (Ramzan et al., 2022). However, we did not find much evidence that has investigated the relationship between ICT diffusion and green growth. In light of the aforementioned discussion, we notice that not many studies have investigated the impact of renewable energy transitions, higher education, and ICT diffusion on environmental sustainability and green growth. To fill this gap in the literature, we endeavor to examine the impact of renewable energy transitions, higher education, and ICT diffusion on environmental sustainability and green growth.

## Literature review

Renewable energy is a cleaner source of energy that leads to environmental sustainability. Renewable energy consumption guarantees energy security that reduces CO_2_ emissions (Thangavelu et al., 2015). To control environmental pollution, economies are converging toward eco-friendly energy technologies (Ullah et al., 2021b). Renewable energy consumption is sustainable, and its price is relatively less volatile than the price of fossil fuel energy sources (Barbir, 2009; Pata, 2021a,b). Global warming and environmental degradation are instigating climatic variations that can be controlled through renewable energy transition (Isik et al., 2018). Various studies have reported the environmental protective role of renewable energy consumption (Panwar et al., 2011; Pata, 2018; Nathaniel and Iheonu, 2019; Sohail et al., 2021; Yuping et al., 2021). Hence, it is confirmed from prior literature that the renewable energy transition exerts a positive influence on environmental quality.

The article "Pro-environmental behavior–Renewable energy transitions nexus: Exploring the role of higher education and information and communications technology diffusion" was retracted in 2025. Reasons: an official misconduct investigation; compromised peer review; a compromised editor; unreliable results or conclusions.

No doubt, education is considered an important determinant that raises knowledge and awareness of people regarding energy efficiency and efficient utilization of energy sources. In this regard, the studies carried out by Liu et al. (2022) in China are found fundamental as these studies have identified two opposing impacts of the educational level on environmental performance. Societies with low education and awareness levels consume more of fossil fuel energy sources and raise the level of CO_2_ emissions (Zhu et al., 2021). By contrast, highly educated and more knowledgeable people reduce the consumption of fossil fuel energy and prefer to use renewable energy sources, thus playing an important role in defining the environmental quality. The CO_2_ emission level can decrease by the adoption of renewable energy sources, environmental regulations, and social awareness in household activities, transport, and workplaces (Sohail et al., 2021). This reveals the significant role of education in the reduction of CO_2_ emissions by augmenting energy security and efficiency.

Another determinant that can play a fundamental role in improving environmental quality is ICT diffusion. Empirical studies exploring the nexus between ICT and environmental performance are extensively growing. Various proxies have been adopted to capture the role of ICT diffusion and environmental quality (Chien et al., 2021). Haini (2021) highlighted that the effect of ICT on environmental quality differs due to the degree of education in society. It is proposed that education augments the usefulness of ICT diffusion in society by enhancing economic absorption abilities. The role of education in facilitating and spreading knowledge regarding ICT diffusion is substantial (Li et al., 2022b). Usman et al. (2021) indicated that education accompanied with ICT diffusion maintains environmental performance by raising awareness about environmental issues and stimulating energy recycling and conservation practices. Some studies reveal that education might suppress or promote the potential effect of ICT diffusion on the environment (Wei and Ullah, 2022). Recent research on the nexus between the environment and ICT diffusion provides mixed findings.

The article "Pro-environmental behavior–Renewable energy transitions nexus: Exploring the role of higher education and information and communications technology diffusion" was retracted in 2025. Reasons: an official misconduct investigation; compromised peer review; a compromised editor; unreliable results or conclusions.

Many professionals and experts denote that green growth is an important determinant for sustainable growth and devise many strategies to achieve green growth. It is argued that eco-friendly energy innovation helps in the attainment of sustainable green growth (Dai et al., 2016). The technologies, equipment, and product that are developed and produced with the efficient and sustainable use of renewable energy sources exert relatively less pressure on environmental performance. Likewise, renewable energy consumption helps guard and preserves the ecological balance by reducing CO_2_ emission levels. Sohag et al. (2021) denoted that developing renewable energy sources may positively influence green growth. Indeed, the renewable energy sector development has become fundamental for the achievement of green growth in any economy. Education and green growth are closely associated with each other (Li et al., 2022b). Wang and Shao (2019) denoted that education can develop long-term green growth as it augments the training and skills of labor force, which is basic input in the production function. The advanced economies have converted their techniques of production that help in the achievement of sustainable green growth (Batool et al., 2019; Li and Ullah, 2022a). Some studies have argued that ICT development can also positively contribute to green growth. The transformation of the economic structure toward ICT development can allow economies to substitute checkbooks, compact disks, books with MP3s, and bytes, which can convert the economic system to be more capital-free and improve economic development (Gao et al., 2022).

Despite the importance of renewable energy transition, ICT development, and education in defining environmental performance and green growth, very limited studies explored this nexus. Most specifically, very rarely studies are conducted on exploring this nexus in China. Moreover, existing literature outlines mixed and inconclusive findings. This research will identify the favorable effect of the renewable energy transition, ICT diffusion, and education on green growth and CO_2_ emissions in China. This study will help policymakers in devising a comprehensive strategy for enhancing green growth and reducing CO_2_ emissions.

## Models and methodology

Following Li et al. (2022b), this study assumes that renewable energy consumption, ICT diffusion, and higher education are significant determinants of green growth and environmental sustainability. The existing studies on environmental performance and green growth have used traditional estimation techniques; however, none of the studies has used the newly developed quantile ARDL approach for making empirical inferences. Thus, to examine the cointegration association between dependent and independent variables, our study has used the QARDL technique. The quantile regression approach has several advantages that make its findings more robust and not influenced by extreme data and abnormal data (Sharif et al., 2020a,b). This technique allows examining the long-run relationship simultaneously with short-term relationships for all quantiles of the concerned variables (Godil et al., 2020). This technique is constructed by Cho et al. (2015) who indicated that the QARDL approach allows for exploring the quantile long-run equilibrium effect of the renewable energy transition, ICT, and education on green growth and environmental sustainability. The long-run relationship among variables is also confirmed through the Wald test, which allows confirming the constancy of coefficients across quantiles. Thus, the equation for the ARDL model can be written as follows:


(1) $${\text{Y}}_{\text{t}}=\mu +\sum_{\text{i}=1}^{\text{p}}\sigma_{{\text{Y}}_{\text{i}}}{\text{Y}}_{\text{t-i}}+\sum_{\text{i}=0}^{\mathrm{n1}}\sigma_{{\text{REC}}_{\text{i}}}\,{\text{REC}}_{\text{t-i}}+\sum_{\text{i}=0}^{\mathrm{n2}}\sigma_{{\text{ICT}}_{\text{i}}}\,{\text{ICT}}_{\text{t-i}}+\sum_{\text{i}=0}^{\mathrm{n3}}\sigma_{{\text{HE}}_{\text{i}}}\,{\text{HE}}_{\text{t-i}}+\sum_{\text{i}=0}^{\mathrm{n4}}\sigma_{{\text{FD}}_{\text{i}}}\,{\text{FD}}_{\text{t-i}}+\varepsilon_{\text{t}}$$

where ε_t_ represents the error term, which is measured through Y_*t*_ -E[Yt/Ft-1], where Ft–1 is the smallest σ-field made by (Y_*t*–1_, REC_*t*_, ICT_*t*_, HE_*t*_, FD_*t*_, Y_*t*–1_, REC_*t*–1_, ICT_*t*–1_, HE_*t*–1_, FD_*t*–1_), and p and n1….n4 signify the lag orders for concern variables, respectively. In addition, in Eq. (1), we confer that renewable energy consumption, higher education, ICT diffusion, and financial development are signified by REC_*t*_, ICT_*t*_, HE_*t*_, and FD_*t*_, respectively, while Y_*t*_ represents a vector of CO_2_ emissions and green growth. Following Cho et al. (2015), the quantile ARDL can be stated in equation (2), respectively:


(2) $${\text{Q}}_{{\text{Y}}_{\text{t}}}=\mu \,\left(\tau \right)+\sum_{\text{i}=1}^{\text{p}}\sigma_{{\text{Y}}_{\text{i}}}\,\left(\tau \right)\;{\text{Y}}_{\text{t-i}}+\sum_{\text{i}=0}^{\mathrm{n1}}\sigma_{{\text{REC}}_{\text{i}}}\,\left(\tau \right)\,{\text{REC}}_{\text{t-i}}+\sum_{\text{i}=0}^{\mathrm{n2}}\sigma_{{\text{ICT}}_{\text{i}}}\,\left(\tau \right)\;{\text{ICT}}_{\text{t-i}}+\sum_{\text{i}=0}^{\mathrm{n3}}\sigma_{{\text{HE}}_{\text{i}}}\,\left(\tau \right)\,{\text{HE}}_{\text{t-i}}\;++\sum_{\text{i}=0}^{\mathrm{n4}}\sigma_{{\text{FD}}_{\text{i}}}\left(\tau \right)\;{\text{FD}}_{\text{t-i}}+\varepsilon_{\text{t }}\left(\tau \right)$$

where εt(τ) = Yt-QYt(τ/Ft-1), and QYt(τ/Ft-1) and 0 >τ< 1 show quantile. To eliminate serial correlation, we have stated equation (2) in the generalized form given as follows:


(3) $${\text{Q}}_{\Delta \,{\text{Y}}_{\text{t}}}=\mu +\rho \,{\text{Y}}_{t-1}+\pi_{\text{REC}}\,{\text{REC}}_{t-1}+\pi_{\text{ICT}}{\text{ICT}}_{t-1}+\pi_{\text{HE}}\,{\text{HE}}_{t-1}+\pi_{\text{FD}}\,{\text{FD}}_{t-1}+\sum_{\text{i}=1}^{\text{p}}\sigma_{{\text{Y}}_{\text{i}}}\,\Delta \,{\text{Y}}_{\text{t-i}}+\sum_{\text{i}=0}^{\mathrm{n1}}\sigma_{{\text{REC}}_{\text{i}}}\,\Delta \,{\text{REC}}_{\text{t-i}}+\sum_{\text{i}=0}^{\mathrm{n2}}\sigma_{{\text{ICT}}_{\text{i}}}\,\Delta \,{\text{ICT}}_{\text{t-i}}+\sum_{\text{i}=0}^{\mathrm{n4}}\sigma_{{\text{HE}}_{\text{i}}}\,\Delta \,{\text{HE}}_{\text{t-i}}+\sum_{\text{i}=0}^{\mathrm{n5}}\sigma_{{\text{FD}}_{\text{i}}}\,\Delta \,{\text{FD}}_{\text{t-i}}+\varepsilon_{\text{t}}\,\left(\tau \right)$$

With the help of model (3), we can state that the probability of contemporaneous correlation between ε_t_ and ΔREC_*t*_, ΔICT_*t*_, ΔHE_*t*_, and ΔFD_*t*_ increases. On the other hand, through the projection of ε_t_ on ΔREC_*t*_, ΔICT_*t*_, ΔHE_*t*_, and ΔFD_*t*_ with the form ε_*t*_ = σ_REC_ΔREC_*t*_+σ_ICT_ΔICT_*t*_+σ_HE_ΔHE_*t*_+σ_FD_ΔFD_*t*_+υ_*t*_, we can eliminate previous correlations. In the next step, we have stated generalized Eq. (3) and reformulated it into the QARDL-ECM version as follows:


$${\text{Q}}_{\Delta \,{\text{Y}}_{\text{t}}}$$

$$=\mu \left(\tau \right)+\rho \left(\tau \right)({\text{Y}}_{\text{t}-1}-\eta_{\text{REC}}\left(\tau \right){\text{REC}}_{\text{t}-1}-\eta_{\text{ICT}}\left(\tau \right){\text{ICT}}_{\text{t}-1}\;+\;\eta_{\text{HE}}\left(\tau \right){\text{HE}}_{\text{t}-1}+\eta_{\text{FD}}\left(\tau \right){\text{FD}}_{\text{t}-1})\;+\sum {}^{\text{p}}{}_{\text{i}=1}\pi {}_{{\text{Y}}_{\text{i}}}(\tau )\Delta \text{Y}{}_{\text{t}-\text{i}}\;+\sum_{\text{i}=0}^{\mathrm{n1}}\pi_{{\text{REC}}_{\text{i}}}\,\left(\tau \right)\,\Delta \,{\text{REC}}_{\text{t}-\text{i}}\;+\sum_{\text{i}=0}^{\mathrm{n2}}\pi_{{\text{ICT}}_{\text{i}}}\,\left(\tau \right)\,\Delta \,{\text{ICT}}_{\text{t}-\text{i}}$$

(4) $$+\sum_{\text{i}=0}^{\mathrm{n3}}\pi_{{\text{HE}}_{\text{i}}}\,\left(\tau \right)\,\Delta \,{\text{HE}}_{\text{t}-\text{i}}\;+\sum_{\text{i}=0}^{\mathrm{n4}}\pi_{{\text{FD}}_{\text{i}}}\,\left(\tau \right)\,\Delta \,{\text{FD}}_{\text{t}-\text{i}}\;+\;\varepsilon_{\text{t}}\,\left(\tau \right)$$

From Eq. (4), we can capture short-run dynamics through π*⁢∑j=1pπj, while long-run cointegration among the variables of renewable energy consumption, higher education, ICT diffusion, and financial development is expressed with the help of $\lambda_{\text{REC}}^{*}\,=-\frac{\lambda \,\text{REC}}{\text{p}},\lambda_{\text{ICT}}^{*}\,=-\frac{\lambda \,\text{ICT}}{\text{p}},\lambda_{\text{HE}}^{*}\,=-\frac{\lambda \,\text{HE}}{\text{p}}$, and $\lambda_{\text{FD}}^{*}\,=-\frac{\lambda \,\text{FD}}{\text{p}}$, correspondingly. The delta technique is useful in measuring different parameters, for instance, long-term cointegration parameters and current and previous parameters. The coefficient (ρ) should be significant and negative. Last, the asymmetric influence of concern variables can be examined through the application of the Wald test.

The article "Pro-environmental behavior–Renewable energy transitions nexus: Exploring the role of higher education and information and communications technology diffusion" was retracted in 2025. Reasons: an official misconduct investigation; compromised peer review; a compromised editor; unreliable results or conclusions.

## Data

To examine the impact of renewable energy consumption, ICT, and education on environmental benefits and green growth, time series data have been collected for the period 1996–2020. The data span is limited from 1996 to 2020 due to the unavailability of data. Table 1 shows detail about the symbols of variables, sources, and definitions. CO_2_ emission (CO_2_) and green growth (GG) are dependent variables in this study. However, renewable energy consumption (REC), ICT, and higher education (HE) are the main independent variables. Financial development (FD) is added as a control determinant in regression analysis. The annual data for all these variables have been collected from various sources, such as WDI, OECD, and IMF. After collecting annual data series, these series are transformed into quarterly data series. This transformation is required for the application of the QARDL regression technique. Transformation of data is performed by using the match sum approach that is developed by Sharif et al. (2019).

**TABLE 1:** Definitions and data sources.

Symbol	Variables	Definitions	Sources
CO_2_	CO_2_ emissions	CO_2_ emissions (kt)	WDI
GG	Green growth	Pollution-adjusted GDP growth (%)	OECD
REC	Renewable energy consumption	Renewable energy consumption (% of total final energy consumption)	WDI
ICT	Information and communications technology	Individuals using the Internet (% of population)	WDI
HE	Higher education	School enrollment, tertiary (% gross)	WDI
FD	Financial development	Financial development index	IMF

## Empirical results

This study intends to explore the nexus among CO_2_ emission, green growth, renewable energy consumption, ICT, higher education, and financial development in China. Table 2 reports the descriptive statistics of all these variables, namely, CO_2_, GG, REC, ICT, HE, and FD in China. Mean values for all the variables are positive. The average value for CO_2_ is 15.67, with 16.33 and 14.93 as maximum and minimum ranges. The mean value for GG is 8.697, with a maximum value of 13.49 and a minimum value of 6.923. The mean of REC is reported 2.823, with a maximum value of 3.423 and a minimum value of 1.498. The average value for HE is 3.002, with 4.104 and 1.562 as maximum and minimum ranges, respectively. The mean value for ICT is 2.150, with a maximum value of 4.292 and a minimum value of −4.514. The mean of FD is reported as 0.497, with a maximum value of 0.675 and minimum value of 0.342. In addition, the findings of the Jarque–Bera test describe that CO_2_, GG, HE, ICT, and FD are statistically significant, confirming that these series are not normally distributed, which confirms that the QARDL approach can be adopted for further analysis (Batool et al., 2019; Mishra et al., 2019). Table 3 describes the results for DF-GLS and PP unit root tests. The outcome of both tests reveals that only HE is I(0) stationary series, and CO_2_, GG, REC, and ICT are I(1) stationary series.

The article "Pro-environmental behavior–Renewable energy transitions nexus: Exploring the role of higher education and information and communications technology diffusion" was retracted in 2025. Reasons: an official misconduct investigation; compromised peer review; a compromised editor; unreliable results or conclusions.

**TABLE 2:** Descriptive statistics.

	Mean	Median	Maximum	Minimum	Std. Dev.	Skewness	Kurtosis	Jarque-Bera	Probability
CO_2_	15.67	15.78	16.33	14.93	0.474	–0.401	1.566	11.25	0.004
GG	8.697	8.295	13.49	6.923	1.328	1.945	6.780	122.5	0.000
REC	2.823	2.671	3.423	1.498	0.418	–0.011	2.598	0.677	0.713
HE	3.002	3.029	4.104	1.562	0.768	–0.403	2.043	6.526	0.038
ICT	2.150	3.121	4.292	–4.514	2.354	–1.460	4.243	41.94	0.000
FD	0.497	0.515	0.675	0.342	0.101	0.103	1.597	8.376	0.015

**TABLE 3:** Unit root test results.

	DF-GLS			PP		
	I (0)	I (1)	Decision	I (0)	Break date	Decision
CO_2_	0.489	−1.689*	I(1)	–0.725	−2.752*	I(1)
GG	0.125	−1.725*	I(1)	–2.324	−5.185***	I(1)
REC	0.925	−1.785*	I(1)	0.321	−2.657*	I(1)
HE	−2.012**		I(0)	−2.789*		I(0)
ICT	−0.625	−1.897*	I(1)	–1.325	−4.365***	I(1)
FD	1.254	−1.785*	I(1)	0.087	−5.366***	I(1)

***p<0.01.

**p<0.05.

*p<0.1.

Table 4 reports the QARDL estimates of the CO_2_ emissions model for China. The ECM term is reported as significantly negative at all quantiles, confirming the dependency of all the parameters. Moreover, the constant term is also found significant at all quantiles. The results in Table 4 reported the long- and short-term association between a dependent variable (CO_2_) and independent variables (REC, HE, ICT, and FD). The long-run parameters are depicted by η, while the short-run parameters are represented by π. The finding of REC shows that it is significantly negative at quantiles 0.20 to 0.95. This finding reveals that REC is negatively associated with CO_2_, which means that an increase in REC will decrease CO_2_. These results are backed by various previous studies (Lei et al., 2022).

The article "Pro-environmental behavior–Renewable energy transitions nexus: Exploring the role of higher education and information and communications technology diffusion" was retracted in 2025. Reasons: an official misconduct investigation; compromised peer review; a compromised editor; unreliable results or conclusions.

**TABLE 4:** QARDL estimates of CO_2_ emissions.

	Constant	ECM	Long-run coefficient				Short-run coefficient				
	μ (τ)	ρ (τ)	η_R*EC*_ (τ)	η_H*E*_ (τ)	η_I*CT*_ (τ)	η_F*D*_ (τ)	π_R*EC*0_ (τ)	π_R*EC*1_ (τ)	π_H*E*_ (τ)	π_I*CT*_ (τ)	π_F*D*_ (τ)
0.05	−8.852***	−0.812***	−0.078	−0.355***	−0.018	1.796***	−0.119***	−0.116***	0.001	0.001	0.026
	(−4.721)	(−7.712)	(−1.239)	(−5.231)	(−1.412)	(7.342)	(−7.549)	(−4.398)	(0.265)	(0.928)	(0.883)
0.10	−9.000***	−0.830***	−0.105	−0.362***	−0.017	1.637***	−0.141***	−0.120***	0.030	0.005	0.108***
	(−9.784)	(−6.380)	(−1.539)	(−5.083)	(−1.338)	(6.409)	(−6.189)	(−3.987)	(1.479)	(1.266)	(2.947)
0.20	−10.90***	−0.765***	−0.333***	−0.164***	−0.003	0.667***	−0.116***	−0.096***	0.011	0.002	0.081***
	(−9.411)	(−7.271)	(−18.25)	(−9.657)	(−0.844)	(6.768)	(−10.51)	(−4.632)	(1.283)	(1.576)	(2.862)
0.30	−11.93***	−0.820***	−0.437***	−0.161***	−0.002	0.657***	−0.120***	−0.111***	0.008	0.001	0.049*
	(−9.524)	(−7.145)	(−18.31)	(−8.969)	(−0.435)	(6.177)	(−10.50)	(−4.986)	(1.181)	(0.886)	(1.728)
0.40	−12.84***	−0.835***	−0.525***	−0.178***	−0.004	0.697***	−0.122***	−0.123***	0.005	0.000	0.033
	(−7.194)	(−6.801)	(−15.63)	(−8.773)	(−1.021)	(5.130)	(−7.297)	(−4.116)	(0.911)	(0.399)	(1.016)
0.50	−13.63***	−0.822***	−0.685***	−0.180***	−0.003	0.899***	−0.119***	−0.116***	0.001	0.001	0.026
	(−7.994)	(−7.712)	(−13.92)	(−8.293)	(−0.723)	(5.720)	(−7.549)	(−4.398)	(0.265)	(0.928)	(0.883)
0.60	−14.42***	−0.779***	−0.639***	−0.199***	−0.002	0.950***	−0.123***	−0.117***	−0.001	0.001	0.033
	(−7.504)	(−7.062)	(−13.64)	(−8.039)	(−0.526)	(6.694)	(−4.633)	(−2.826)	(−0.115)	(1.273)	(1.035)
0.70	−16.37***	−0.732***	−0.628***	−0.186***	−0.001	1.077***	−0.121***	−0.108***	−0.007	0.003	0.019
	(−9.574)	(−5.232)	(−15.71)	(−6.677)	(−0.118)	(7.468)	(−6.607)	(−2.923)	(−0.780)	(1.255)	(0.474)
0.80	−16.35***	−0.616***	−0.629***	−0.193***	−0.015	1.111***	−0.141***	−0.101*	−0.012	0.004**	0.008
	(−9.225)	(−7.778)	(−18.18)	(−5.372)	(−0.059)	(6.968)	(−3.224)	(−1.742)	(−1.356)	(2.534)	(0.184)
0.90	−16.22***	−0.656***	−0.608***	−0.236***	−0.096**	1.054***	−0.193	−0.095	−0.019	0.006**	0.061
	(−8.634)	(−3.314)	(−15.05)	(−5.312)	(−2.019)	(4.432)	(−1.599)	(−1.371)	(−1.029)	(2.424)	(1.191)
0.95	−15.98***	−0.572***	−0.566***	−0.259***	−0.110**	1.201***	−0.261*	−0.082	−0.003	0.003*	0.055
	(−7.051)	(−3.056)	(−20.74)	(−8.566)	(−2.212)	(7.176)	(−1.926)	(−1.115)	(−0.183)	(1.826)	(0.851)

The table reports the quantile estimation results.

***p<0.01.

**p<0.05.

*p<0.1.

The article "Pro-environmental behavior–Renewable energy transitions nexus: Exploring the role of higher education and information and communications technology diffusion" was retracted in 2025. Reasons: an official misconduct investigation; compromised peer review; a compromised editor; unreliable results or conclusions.

The HE effect is found significantly negative at all quantiles. This result specifies that at all quantiles, an increase in HE decreases CO_2_ in China. This outcome is aligned with the results of the study carried out by Li and Ullah (2022b). Moreover, Jian et al. (2021) indicated that higher education can effectively result in the mitigation of CO_2_ emissions. The ICT is found significant and negative at higher quantiles only, that is, 0.90 and 0.95. This result shows that an upsurge in ICT reduces CO_2_ emissions in China at higher intensities only. Usman et al.’s (2022) study also reported a similar negative relationship between CO_2_ and ICT. The outcome of FD indicates that it is significantly positive at all quantiles. It means that an increase in the FD increases CO_2_ emissions in China. A similar nexus between FD and CO_2_ is reported by Li et al. (2022a). The short-run findings describe that the REC impact on CO_2_ emissions is reported significantly negative at all quantiles, except 0.90. However, the HE impact on CO_2_ is reported insignificant at all quantiles. ICT reports a significantly positive impact on CO_2_ emissions at higher quantiles only, that is, 0.80 to 0.95.

Table 5 reports the QARDL estimates of the green growth model for China. The ECM term is found significantly negative at all quantiles. Moreover, the constant term is also reported significant at all quantiles. Table 5 displays the long-and short-term relationship between a dependent variable (GG) and independent variables (REC, HE, ICT, and FD). The finding of REC shows that it is significantly positive at quantiles 0.50 to 0.95. This finding reveals that REC is positively associated with GG, which shows that in China, an increase in REC will increase GG. These results are supported by various previous studies (e.g., Gu et al., 2018).

**TABLE 5:** QARDL estimates of green growth.

	Constant	ECM	Long-run coefficient				Short-run coefficient				
	μ (τ)	ρ (τ)	η_R*EC*_ (τ)	η_H*E*_ (τ)	η_I*CT*_ (τ)	η_F*D*_ (τ)	π_R*EC*_ (τ)	π_H*E*_ (τ)	π_I*CT*_ (τ)	π_F*D*0_ (τ)	π_F*D*1_ (τ)
0.05	4.109**	−0.459**	0.171	2.999***	0.213***	1.235***	0.574***	1.541	0.064	1.518	0.927***
	(2.511)	(−2.104)	(0.538)	(5.206)	(6.594)	(3.785)	(3.761)	(0.524)	(0.617)	(0.093)	(2.769)
0.10	5.371***	−0.479**	0.199	2.940***	0.234***	1.654***	0.342***	2.363	0.143	1.654	1.044***
	(3.328)	(−2.138)	(0.016)	(4.857)	(5.893)	(4.099)	(2.665)	(0.798)	(1.581)	(0.989)	(3.735)
0.20	6.469***	−0.542**	0.231	2.088***	0.321***	1.987***	0.191***	0.581	0.013	1.987***	0.484***
	(3.588)	(−2.230)	(0.063)	(3.088)	(3.120)	(2.946)	(2.814)	(0.285)	(0.371)	(2.587)	(6.051)
0.30	6.665***	−0.564**	0.258	2.364***	0.345***	2.325***	0.181**	1.840	0.002	2.321*	0.519***
	(2.723)	(−2.044)	(0.284)	(3.167)	(3.989)	(2.818)	(2.441)	(0.741)	(0.036)	(1.842)	(4.172)
0.40	7.658***	−0.589**	0.287	1.595**	0.399***	2.654***	0.161**	1.907	0.004	2.542***	0.532***
	(3.175)	(−2.243)	(1.555)	(2.571)	(4.015)	(2.938)	(2.078)	(0.834)	(0.101)	(2.643)	(3.257)
0.50	8.654***	−0.621***	0.321**	1.056*	0.412***	2.789**	0.178*	1.870	0.022	2.875***	0.519**
	(4.435)	(−2.623)	(2.116)	(1.664)	(3.128)	(2.308)	(1.724)	(0.887)	(0.610)	(2.864)	(2.516)
0.60	9.654***	−0.645**	0.354***	1.345**	0.456*	2.987*	0.198*	2.211	0.057*	2.954*	0.404***
	(5.130)	(−2.283)	(2.595)	(2.304)	(1.771)	(1.743)	(1.775)	(1.068)	(1.726)	(1.783)	(3.414)
0.70	10.23***	−0.721**	0.452***	1.654**	0.542**	3.214***	0.177*	2.218	0.063**	3.215*	0.384***
	(5.011)	(−2.024)	(2.837)	(2.325)	(2.253)	(2.960)	(1.686)	(1.150)	(2.191)	(1.828)	(7.279)
0.80	11.23***	−0.754**	0.542***	1.987***	0.654**	3.425***	0.213	1.044	0.062*	3.354	0.400***
	(6.713)	(−2.179)	(4.390)	(2.654)	(2.439)	(3.858)	(1.630)	(0.574)	(1.889)	(0.305)	(7.224)
0.90	13.21***	−0.775**	0.654***	2.012***	0.758*	3.456	0.254	0.698	0.193**	3.487	0.523***
	(3.365)	(−2.193)	(2.757)	(2.020)	(1.958)	(1.519)	(1.570)	(0.408)	(2.545)	(0.362)	(6.442)
0.95	14.36***	−0.795**	0.745***	2.321***	0.894**	3.564	0.298	1.132	0.226***	3.542	0.600***
	(3.765)	(−2.394)	(2.930)	(3.077)	(2.152)	(1.508)	(1.289)	(0.484)	(2.846)	(0.316)	(4.864)

The table reports the quantile estimation results.

***p<0.01.

**p<0.05

*p<0.1.

The article "Pro-environmental behavior–Renewable energy transitions nexus: Exploring the role of higher education and information and communications technology diffusion" was retracted in 2025. Reasons: an official misconduct investigation; compromised peer review; a compromised editor; unreliable results or conclusions.

The HE effect is found significantly positive at all quantiles. This result stipulates that at all quantiles, an increase in HE increases GG in China. This outcome is in line with the study carried out by Li et al. (2022b) who denoted that a higher level of education tends to enhance green growth. ICT is found significant and positive at all quantiles in China. This result shows that an upsurge in ICT enhances GG in China at all intensities. Li et al. (2022b) reported a similar positive connotation between GG and ICT. The outcome of FD indicates that it is significantly positive at all quantiles, except 0.90 and 0.95. It means that an increase in the FD enhances GG in China. A similar nexus between FD and GG is reported by Cao et al. (2022). The short-run findings define that the REC impact on GG is reported significantly positive at all quantiles, except 0.80 to 0.95. Conversely, the HE impact on GG is reported insignificant at all quantiles. ICT reports a significantly positive impact on GG at selected quantiles, that is, from 0.60 to 0.95. In Table 6, the Wald test also reported the consistency of the empirical results.

**TABLE 6:** Wald test result.

Variable	CO_2_ emissions			Green growth	
	Wald-stat	Prob.	Variable	Wald-stat	Prob.
ρ	3.046***	0.000	ρ	3.459***	0.000
η_REC_	5.658***	0.000	η_REC_	6.117***	0.000
η_HE_	4.239***	0.003	η_HE_	6.201***	0.003
η_ICT_	1.018	0.210	η_ICT_	1.028	0.200
η_FD_	3.897**	0.018	η_FD_	2.897**	0.021
π_*REC0*_	4.021***	0.005	π_REC_	0.010	0.966
π_*REC1*_	1.035	0.694	π_HE_	2.165	0.624
π_HE_	1.003	0.829	π_ICT_	0.004	0.971
π_ICT_	1.001	0.667	π_*FD0*_	7.315***	0.002
π_FD_	0.064	0.380	π_*FD1*_	4.252***	0.001

***p<0.01.

**p<0.05.

*p<0.1.

The article "Pro-environmental behavior–Renewable energy transitions nexus: Exploring the role of higher education and information and communications technology diffusion" was retracted in 2025. Reasons: an official misconduct investigation; compromised peer review; a compromised editor; unreliable results or conclusions.

## Results and discussion

The study confirms that to reduce carbon emissions and achieve green economic growth, a transition to renewable energy is essential. There is a consensus among policymakers, empirics, and environmentalists that renewable energy consumption is the most feasible option to tackle the problem of environmental degradation and carbon-packed economic growth (Li and Ullah, 2022b). Renewable energy sources are the zero-carbon sources of energy that are crucial for the sustainable future of the world. Therefore, the departure from non-renewable energy sources and the adoption of renewable energy sources are of paramount importance for separating economic growth and CO_2_ emissions (Maji, 2019). These findings are supported by the decisions taken by the international community in various instances, such as the United Nations Agenda for Sustainable Development 2030 and the Paris Agreement 2015 (Fuso Nerini et al., 2018). Renewable energy transition helps protect the environment and enhance green growth. Our findings are backed by Ackah and Kizys (2015) who noted that renewable energy can mitigate CO_2_ emissions through modification of the energy sector that enhances green growth. Moreover, environmental pressures have stimulated the renewable energy demand, which led to enhanced renewable energy capacity, which, in turn, upsurges green growth (Sohag et al., 2021).

Other significant findings of the study confirm the positive impact of ICT on green growth and the negative impact on CO_2_ emissions. According to Li et al. (2022b), promoting electronics production required software, and services sectors depend on the ICT industry development. The dematerialization and demobilization of the economy can be achieved through increased use of information resources, which would help reduce the burden on the environment without compromising economic targets (Usman et al., 2021). These findings are in line with the guidelines of the European Commission (2006), which state that “ICT plays an important role in reducing energy intensity and increasing the energy efficiency of the economy” (Lange et al., 2020), crucial for improving environmental quality and promoting long-run economic growth. Li et al. (2022b) supported our findings by arguing that ICT development, including full use of disseminated information, openness, sharing, and interaction, can improve and promote environmental sustainability and green growth. Li and Zhao (2021) explained that ICT use reduces the energy intensity in the economy, promotes environmental performance, and ensures green development.

The article "Pro-environmental behavior–Renewable energy transitions nexus: Exploring the role of higher education and information and communications technology diffusion" was retracted in 2025. Reasons: an official misconduct investigation; compromised peer review; a compromised editor; unreliable results or conclusions.

Finally, higher education can bring awareness to society regarding improving environmental quality and is a crucial source for building skilled and trained labor, which is crucial for promoting clean and green manufacturing practices (Ullah et al., 2021a). Therefore, a highly educated society is more likely to achieve sustainable economic development (Wei et al., 2022). Our findings are in line with the findings of Bano et al. (2018). Li et al. (2022b) study highlighted that education helps in the innovation of more efficient energy technologies. Education also contributes to the formation of human capital, which leads to green growth and economic development. Wang and Shao (2019) justified our findings as education empowers society to expand the processes and methods of production to achieve innovation, environmental protection, and green development.

## Conclusion and implications

Climate change and global warming are the major concerns that have irked the international community. According to the available empirical evidence, anthropogenic activities driven by fossil fuels are the leading cause of GHG emissions, resulting in climate change and global warming. Global warming has caused rising sea levels, melting glaciers, frequent floods, tornados, hurricanes, and deterioration in agricultural output, and all these climate problems have threatened the existence of humanity. Therefore, policymakers and academics are in search of the factors that can significantly cut GHG emissions without hindering economic development. The most accepted solution to deal with the problems of global warming and climate change is to transform the energy sector by moving toward renewable energy. Education can increase people’s consciousness about environmental quality and encourage them to increase renewable energy consumption. Similarly, ICT can improve the economy’s technological development, facilitating the renewable energy transition. Therefore, the primary focus of the analysis is to examine the role of renewable energy consumption, higher education, and ICT in improving environmental quality.

For investigating the short- and long-run relationship between renewable energy consumption, higher education, and ICT on CO_2_ emissions and green growth across various quantiles, we have employed the quantile ARDL model. According to the findings of QARDL, the long-run estimated coefficients of renewable energy consumption and higher education are positively significant in most quantiles, signifying the positive contribution of renewable energy consumption and higher education in improving environmental quality. However, in the long run, the estimates attached to ICT are insignificant in the CO_2_ emissions model in most quantiles. On the other hand, the estimates of renewable energy consumption are significantly positive from the 50th quantile onward in the green growth model, confirming that the higher the renewable energy in the economy, closer it will get to the target of green economic growth. The estimates of higher education and ICT are positively significant at most quantiles in the green growth model, implying that both higher education and ICT pave the way for green economic growth in the long run. In the short run, renewable energy consumption turned out to be the most critical determinant of CO_2_ emissions and green growth. Furthermore, the asymmetric impact of renewable energy consumption, higher education, and ICT on CO_2_ emissions and green growth can be seen through significant WALD statistics in both the short and long run.

The article "Pro-environmental behavior–Renewable energy transitions nexus: Exploring the role of higher education and information and communications technology diffusion" was retracted in 2025. Reasons: an official misconduct investigation; compromised peer review; a compromised editor; unreliable results or conclusions.

Based on these findings, we can derive some important policy implications. First, the positive role of renewable energy consumption is confirmed in improving environmental quality and achieving green growth. Therefore, increasing the renewable energy share is the panacea to improving environmental quality and achieving green growth. Hence, policymakers must increase investment in renewable energy technologies and research and development activities that would help increase renewable energy consumption. The potential of the renewable energy sector is not fully explored; thus, it is required to enhance government subsidy for investment in the renewable energy sector that results in a reduction of carbon emissions. Moreover, complete information regarding green investment should be shared with all segments of the economy to achieve green growth. Second, the development of ICT can lead the economy toward a dematerialized and weightless economy, which is crucial for sustainable development. Hence, the transition of the economy from physical to information sources is vital for improving environmental quality without conceding the economic goals. Last, increasing the formal literacy rate can make people aware of the issue of environmental degradation, and they would increase their efforts for the sustainable development of society and the economy.

The article "Pro-environmental behavior–Renewable energy transitions nexus: Exploring the role of higher education and information and communications technology diffusion" was retracted in 2025. Reasons: an official misconduct investigation; compromised peer review; a compromised editor; unreliable results or conclusions.

The present study contains some limitations that need to be addressed in future studies. The present research covers data spanning from 1996 to 2020 due to the unavailability of data before that period. Another limitation is that the study covers the Chinese economy only. In future, researchers must investigate the aforementioned nexus for different regions and countries. The present study only uses green growth and CO_2_ emissions to measure pro-environmental behavior. Future studies can use other measures of pro-environmental behavior. In addition, the use of the NARDL technique can provide more clear evidence regarding the asymmetric relationship between pro-environmental behavior and renewable energy transition. Apart from renewable energy consumption, higher education, and ICT, future studies must include other variables, such as environmental innovations, green investment, and financial inclusion as a determinant of green economic growth.

## Data availability statement

The original contributions presented in this study are included in the article/supplementary material, further inquiries can be directed to the corresponding author/s.

## Author contributions

All authors listed have made a substantial, direct, and intellectual contribution to the work, and approved it for publication.
